# Analysis on the Influencing Factors and Training Strategies of Young Talents in Hospitals under the Background of Big Data

**DOI:** 10.1155/2022/6213592

**Published:** 2022-07-26

**Authors:** Ping Liu, Feng Zhao

**Affiliations:** Tianjin Medical University General Hospital, Tianjin 300052, China

## Abstract

Under the background of big data, young talents in hospitals across my country are constantly striving to exert their personal scientific research and technical capabilities in terms of scientific research performance. At the same time, it also exposed many problems that need to be solved urgently. Under the background of the new era, each hospital needs to exert and increase its training in terms of scientific research and technology research and the use of young talents. By building a scientific platform and establishing an effective scientific research performance evaluation management system, the backbone of outstanding young medical talents can be realized. In the context of big data, this paper studies and analyzes the influencing factors of hospital young talent scientific research and performance management. After the preliminary data collection work, the chi-square verification was carried out on the survey data of young medical scientific research talents. It is confirmed that the research conclusions based on big data have certain basis for improving the scientific research management level of each hospital based on the research conclusions, thus providing a certain theoretical basis for enhancing the scientific research performance of young talents in the hospital.

## 1. Introduction

The new generation of young scientific research talents has an important impact on the hospital's improvement of medical technology level and the expansion of research in the medical field. In recent years, with the continuous development of global medical technology, hospitals have made certain explorations in improving the scientific research and training mechanism of young talents, and hospitals have also provided a large number of scientific research platforms and research channels while paying attention to the training of young talents [1, 2]. However, in the context of the new era, hospitals still need to exert and increase their training efforts in scientific research and technology research and the use of young talents and realize the scientific utilization of outstanding young medical talents by building a scientific platform and establishing an effective scientific research performance evaluation management system [3, 4]. Some scholars have adopted the method of empirical research to investigate the current situation of scientific research of young talents in some hospitals and in-depth analysis of various factors that affect their enthusiasm for scientific research, and based on this, they have constructed a relatively comprehensive talent scientific research promotion plan [5–7].

Based on the investigation and understanding of the scientific research performance of young talents in hospitals, this study studies the influencing factors of the entire hospital scientific research performance industry and conducts research and evaluation analysis on the key directions of subjective influencing factors in the implementation of scientific research performance of young talents, so as to propose targeted improvement and training strategies [8, 9]. Through the data research method based on the conditions of big data technology, the focus is on the comprehensive investigation and understanding of young scientific researchers, including doctors, major talents in various scientific research aspects of medical technology, and scientific research system. Through the analysis and study of the survey data, through statistical analysis, multiple linear regression display, and chi-square verification, the influencing factors of young scientific research talents in the entire medical field are explored and studied in an all-round way, and the improvement measures and methods are targeted and clear [10, 11].

## 2. The Current Situation of the Industry in the Context of Big Data

The development of big data technology has brought a violent impact on the traditional work formats of various industries.

### 2.1. The Basic Understanding of Big Data in Hospital Scientific Research Work

The advent of the information technology era has brought the level of scientific research technology development in various industries to a new level, and the hospital scientific research work in the context of big data has also been greatly improved and innovated, compared to the traditional hospital scientific research work, and the scientific research work in the context of big data can effectively show the great changes brought by the new era to the medical progress of hospital scientific research, through extensive access to sort out big data, in the process of analyzing big data, and fully grasp the shortcomings and deficiencies in the field of medical research [12–15]. Through targeted medical research, the wide application of big data technology is realized, and the wide application of big data in medical research work is enhanced [16, 17]. Through professional data analysis and scientific research technology research, it can effectively improve the work quality and efficiency of hospital scientific research workers, especially the young generation of scientific research workers.

For the young generation of medical research work, in the entire scientific research implementation process, in the context of big data, facing the scientific research business data, attach importance to the collection and collation of relevant data relations, through the acceptance of diversified data changes, through the summary analysis of the survey results, the final research direction of scientific research is formed, and the corresponding medical research predictions and results are obtained, as detailed in Figure 1.

### 2.2. Integration of Big Data and Hospital Youth Performance

The young generation is affected by various factors in the scientific research work of the hospital, and the role of medical research brought by big data and cloud computing cannot be ignored. With the continuous integration and development of new disciplines such as information technology and clinical medicine, the young talents of the hospital in the field of scientific research deepen their cognition and promote development through the rational use of data scale, promote the research depth and field expansion of the entire medical research field, and provide a more solid foundation for the scientific research management and refined and intelligent medical implementation of the entire hospital by making a large amount of medical data and effective, diversified, and high-value [18, 19]. The use of new thinking and new initiatives promotes the progress of the hospital's overall medical research career.

## 3. Hospital Youth Scientific Research Survey under Big Data Statistics

The most critical part of hospital youth scientific research is the mastery of relevant data. With the support of big data technology, this work has been carried out smoothly.

### 3.1. Data Analysis Methods

Through the investigation and understanding of the research performance of hospital youth in the context of big data, based on the research and understanding of the training of young talents and work performance of hospitals, through the use of 5 points of objectives, of which 5 points are scored for complete satisfaction, 4 points for satisfaction, generally 3 points, 2 points for dissatisfaction, and 1 point for complete dissatisfaction, under the premise of big data analysis, 250 young researchers were randomly selected [20, 21]. Real-time data research, on the basis of data analysis, through in-depth interviews and research on mechanisms and systems of hospital researchers at different levels, was as follows. From multiple angles, we will solicit and understand the hospital's suggestions and measures on the performance of young talents in the training of scientific research teams. In order to more effectively validate the research proposal, the study used a 10-fold crossvalidation method to divide the 250 young researchers into 5 groups. One group was randomly selected as the experimental group in each research cycle, and the remaining 4 groups were used as the control group. The group, through the results of multiple experiments, optimizes the research proposal.

### 3.2. Investigation of the Performance of Young Medical Talents in Scientific Research Work

Through the performance satisfaction survey of 250 young workers selected under the background of big data, the average satisfaction value was 3.5. This value is between the more satisfactory and general level, reflecting the scientific research workers in their own development and work platform, the overall development level of the entire industry has a certain deficiency and gap, through the analysis of each data index system, as well as in the research process for the performance return management mechanism, and the satisfaction of the scientific research environment survey, the results show that the overall level of development is low, the standard deviation of satisfaction of each indicator is basically concentrated in about 1, and the degree of satisfaction is better.

### 3.3. Satisfaction Analysis of Young Medical Talents on the Scientific Research Performance Management Mechanism

By analyzing the satisfaction of young talents in hospitals with the scientific research performance management mechanism, the survey results show that in the entire operation of the management mechanism, young hospital workers lack stable funds and technical support for the implementation of scientific research performance and have a large room for progress in terms of sense of belonging and achievement [22–24]. Although most of the researchers were relatively satisfied with the hospital operation and management mechanism, reaching 78%, of course, 22% of the respondents rated it as less than satisfied. In the view of different young workers, the influencing factors for the management of hospital scientific research performance are multifaceted, and in the effective prevention and treatment of these influencing constraints, the means and measures of hospitals are not sound and perfect.

### 3.4. The Scientific Research Performance Evaluation Model of Young Talents in the Hospital Is Established

The distribution function of overall research performance is *f*(*x*). The distribution law of population *X* is *M*{*X* = *x*_*i*_) = *m*_*i*_, *i* = 1, 2, ⋯, by dividing the range of values for the overall *X* of scientific performance into *k* small intervals that do not intersect with each other *ξ*_1_, *ξ*_2_, *ξ*_3_, ⋯, *ξ*_*K*_, as shown in formulas (1)–(2).

(1) $$\begin{array}{c} \xi_{1}=\left(\sigma_{0},\sigma_{1}\right],\xi_{2}=\left(\sigma_{1},\sigma_{2}\right],\cdots ,\xi_{K}=\left(\sigma_{k-1},\sigma_{k}\right], \end{array}$$

(2) $$\begin{array}{c} X^{2}=\overset{k}{\underset{i=1}{\sum }}\frac{{\left(f_{i}-{nm}_{i}\right)}^{2}}{{nm}_{i}}. \end{array}$$

### 3.5. Analysis of the Satisfaction of Young Medical Talents with the Scientific Research Environment

For young medical talents, a good scientific research environment will create a good role in promoting scientific researchers. In the process of engaging in scientific and medical research, satisfactory and relatively satisfied about 61.2% in all of participant, the remaining 38.8% chose the opposite option. It shows that there is still a lot of room for improvement in the hospital's scientific research environment for young workers. Moreover, further improving the scientific research working environment has a very important role in promoting and promoting scientific research workers in medical public relations and medical problem solving [25, 26].

### 3.6. Satisfaction Analysis of Young Medical Talents on Work Returns

In the process of surveying the satisfaction of scientific research returns, the satisfaction of young talents in hospitals with the returns to scientific research work has reached 65% above average, but 35% of youth workers still do not think so. Tables 1–3 reflect that in the process of transforming scientific research work and actual benefits in medical scientific research work, there are still certain institutional defects and insufficient promotion power.

## 4. The Main Factors Affecting the Scientific Research Work of Young People in the Hospital and Countermeasures

Through the analysis of big data, we summarize several main factors that currently affect the scientific research work of young doctors and put forward suggestions for the development of these factors.

### 4.1. Main Factors

#### 4.1.1. Engineering Contradictions Are Prominent

In the process of investigation, it was found that young scientific and technological talents should not only face clinical work pressure in the actual clinical teaching and scientific research work but also bear the pressure of hard indicators of scientific research [27, 28]. Say one word: young physicians have a certain engineering contradiction pressure from daily work and scientific research. Moreover, for a team-based scientific research work, it is necessary to have a sense of responsibility and knowledge collaboration of the team and achieve the realization of the performance and value improvement of the entire team through reasonable capital investment, as shown in Figure 2. It can be seen that the system under the current stage has great pressure on the work and scientific research of young workers.

#### 4.1.2. Insufficient Resources for Scientific Research Projects

For a scientific research work, it is necessary to give the greatest support and assistance in human funds and material investment. Young medical workers, in the actual scientific research work, are often full of passion, active thinking, and more agile thinking, but if subject to the obstruction of scientific research project funding resources, it will greatly weaken the enthusiasm and creativity of their work and have a greater impact on scientific research work [29, 30]. Moreover, in terms of scientific research funds, project approval, funding investment, training, and education, the allocation and support of opportunities and inputs in the hospital are not balanced enough, which greatly hinders and reduces the scientific research enthusiasm of young medical workers and hinders the innovative development of medical research projects.

#### 4.1.3. The Mechanism for Cultivating Young Talents Is Not Sound Enough

The cultivation and teaching of young medical research talents are the most fundamental basis and condition for promoting the long-term development and construction of the scientific research performance of the entire medical system, in the implementation of the major hospitals in the talent training and construction path, medical young scientific research workers in the school after leaving the school's scientific research mentor, but also to establish their own new scientific research thinking, in the process of effective scientific research exploration, and the need for hospitals to establish a training platform to promote and cultivate the young generation of scientific research thinking and exploration spirit, through the combination of effective work experience and all-round test verification, to achieve the continuous improvement of scientific research capabilities [31]. Under the condition that the talents under the current mechanism are under the conditions of greater pressure in work and less opportunities and frequencies for training, the investment in the cultivation of young talents' scientific research ability is insufficient, the development prospects are limited, and the imperfection of the talent mechanism has a greater impact on the construction and long-term development of young doctors' scientific research ability.

#### 4.1.4. The Impact of the Family Environment on Scientific Research Work

For young workers in the primary stage and rising stage of their careers, the energy expenditure on family problems also restricts their energy investment in the field of scientific research to a certain extent, and through the understanding of the survey data, it is found that in the work of the young generation, the pressure brought by their families, as well as the guarantee mechanism given by the hospital in actual work, is not perfect and sound, resulting in the young generation to face both the pressure of life brought by society and life, and the pressure brought by work and scientific research, under the dual pressure, to a certain extent, shares the spiritual and energy investment of young workers, resulting in insufficient energy and energy invested in the field of scientific research, which restricts scientific research innovation and medical research.

### 4.2. Improve the Effective Mechanism for the Scientific Research Ability of Young Talents in Hospitals

For a long time, the hospital still has a lot of room for development in terms of scientific research management and incentive mechanism in the field of scientific research. There is still a large room for development; in the establishment of a relaxed scientific research environment, to create a scientific and reasonable scientific research atmosphere, the establishment of effective punishment mechanism and other aspects of the strength is not enough, through the support and subsidies for the family life of scientific research workers, to achieve scientific research workers can put more energy and ideas into scientific research work innovation and medical topics of the research aspects and to achieve the sustainable development of the entire hospital scientific research level.

#### 4.2.1. Build a Platform to Improve the Talent Management Mechanism

As a management department that guides and promotes the long-term development and encouragement of young talents in the field of scientific research, the hospital should make greater efforts and invest more funds in building a reasonable talent training mechanism, and through continuously expanding the scope of talent selection, starting from the special characteristics of different young people, based on different medical topics, to achieve the cultivation of talents and the accumulation of experience for young workers, the results of the survey can also be better confirmed, in the improvement of the talent training mechanism. It can effectively promote the improvement of the level of medical research in a hospital. Perfect young talents, training management mechanism, are to promote and enhance the hospital young workers to put greater energy and their own creative thinking into scientific research work of the effective guarantee and institutional basis, through the hospital's leadership and thinking guidance, so that more young workers from the beginning of the work form and cultivate scientific research thinking and innovative thinking, in the work to accumulate experience and in the scientific research to enhance the ability.

#### 4.2.2. Improve the Scientific Talent Incentive Mechanism

The hospital's scientific research incentive mechanism has a certain cultural guidance and supervision role for young workers, through the establishment of a stronger incentive environment for young talents, to further improve the efficiency of medical research workers, the hospital in the overall atmosphere and platform construction to invest more human and financial support, and the formation of a good scientific research environment and scientific research platform, through the implementation of the hospital's different levels of selection activities and financial, material and spiritual rewards. Establish a scientific research performance evaluation system, realize the affirmation of individual ability through quantitative scientific research ability evaluation, and create a more fair and reasonable environment for talent training, to effectively supervise and guide young workers to exert greater energy and their own creative thinking into the field of medical research work, which further strengthen the long-term development of the hospital's young talents and their recognition of the entire scientific research environment of the hospital and contribute to the overall construction of the hospital and the level of scientific research development.

Also, they should better play the hospital's talent guarantee mechanism for young scientific research workers, through the policy tendencies and subsidies for the family life of young talents in hospitals, to achieve the care and love for the entire young scientific research team and further enhance the energy investment of scientific research workers in scientific research work and public relations of medical problems. Through the establishment of certain guarantee funds and policy working mechanisms, we can effectively enhance the ability of young workers to innovate in cognition and concepts. A perfect scientific research guarantee mechanism can effectively improve the young scientific research workers in the hospital in the most energetic work, and the most innovative spirit of the age group can better participate in scientific research innovation and medical topic public relation process.

#### 4.2.3. Construct a Talent Echelon Training Pyramid

Through the establishment of a pyramid model based on the cultivation of young talents in hospitals, the long-term development of the entire hospital's young talents is realized, and the selection of the entire medical youth team is realized through the layering of 4 stages. Stage 1 belongs to the enlightenment phase, in which a large number of young talents are introduced, and the classification and screening of people at level 1 are achieved by discovering their expertise and interests in unique fields. The second stage belongs to the development stage. Through the screening of the first stage, young talents are cultivated and excavated in their respective specialties, so as to realize the accumulation of primary experience in the field of scientific research. The third stage belongs to the incubation and training stage, which gives young workers certain scientific research responsibilities and difficult problems in terms of unique scientific research projects and medical problems, and enhances personal scientific research public relations capabilities through the accumulation of practical experience. The fourth stage is the actual combat stage, based on the accumulation of previous experience and ability improvement, through the independent undertaking of certain scientific research problems to achieve full play and excavation of personal ability, as shown in Figure 3.

#### 4.2.4. Build a Good Home Environment

Hospital leaders and trade unions should actively understand the family status of young doctors, carry out mutual assistance and cooperation within their capabilities, and relieve certain back-ups for them to carry out scientific research. Although this does not ensure that their family problems are completely solved, the support and care from colleagues and leaders will definitely become a strong motivation for them to study their business.

## 5. Conclusion

The young generation, especially working in the hospital, is an important force in scientific research and innovation. They have a more active thinking and innovative spirit, but the unit brought by the multifaceted pressure let them actually engage in scientific research and daily work. In this regard, the need for the society and hospital groups in the work was as follows: to give them greater help and support, to be more protective of their innovation enthusiasm and initiative, and to cultivate their courage to innovate, the courage to take responsibility of the spirit of scientific research. These tasks are indeed difficult in the past technical background, but at this stage, thanks to the development of Internet of Things technology, young researchers can collect data and conduct experimental observations through the reasonable installation of sensors. Research shows that the application of IoT technology can reduce the average data collection time and experiment cycle by 30%, while the accuracy rate can be improved by more than 15%. So, in a good scientific research environment, they can keep improving the guarantee mechanism. Hospital have to promote the long-term construction of the medical youth work team, establish a scientific research platform suitable for different outstanding young talents, cooperate with advanced medical institutions at home and abroad to cultivate and jointly tackle key problems, and achieve the improvement of the overall scientific research level of the hospital. In the next research, the research will select several representative hospitals, according to their current situation in the construction of young scientific and technological talents team, combined with the conclusions drawn in this study, to build a young scientific talent training system that is more in line with the actual needs of grassroots hospitals.

## Figures and Tables

**Figure 1:** Application process of big data for scientific research data.

**Figure 2:** Mechanism model of team capital investment on team innovation performance.

**Figure 3:** Pyramid model of scientific research ability training of young talents in hospitals.

**Table 1:** Survey on the satisfaction of medical youth with the management mechanism of scientific research performance.

Project	Frequency	Theoretical proportion
Totally satisfied	42	16.8%
Satisfied	66	26.4%
So-so	60	24%
Less satisfied	47	18.8%
Dissatisfied	35	14%
Total	250	100%

**Table 2:** Satisfaction analysis of young medical talents with the working environment.

Project	Frequency	Theoretical proportion
Totally satisfied	45	18%
Satisfied	69	27.6%
So-so	46	18.4%
Less satisfied	50	20%
Dissatisfied	40	16%
Total	250	100%

**Table 3:** Satisfaction analysis of young medical talents with scientific research returns.

Project	Frequency	Theoretical proportion
Totally satisfied	23	9.2%
Satisfied	49	19.6%
So-so	56	22.4%
Less satisfied	62	24.8%
Dissatisfied	60	24%
Total	250	100%

## Data Availability

The data used to support the findings of this study are available from the corresponding author upon request.
